The article "High doses of garlic extract significantly attenuated the ratio of serum LDL to HDL level in rat-fed with hypercholesterolemia diet" was retracted in 2016. Reasons: plagiarism; compromised peer review; false authorship; unreliable data.

# High doses of garlic extract significantly attenuated the ratio of serum LDL to HDL level in rat-fed with hypercholesterolemia diet

**DOI:** 10.1186/s13000-015-0322-0

**Published:** 2015-06-20

**Authors:** Tahereh Ebrahimi, Behnoosh Behdad, Maryam Agha Abbasi, Rahman Ghaffarzadegan Rabati, Amir Farshid Fayyaz, Vahid Behnod, Ali Asgari

**Affiliations:** Department of Agricultural Biotechnology, Sari Agricultural Sciences and Natural Resources University, Sari, Iran; Shahid Beheshti University of Medical Sciences, Tehran, Iran; Department of Biochemistry, College of Science, Kurdistan Science and Research Branch, Islamic Azad University, Sanandaj, Iran; Danesh Pathobiology Laboratory, Tehran, Iran; Shahid Abbas Abdollahi, Molecular Biology Research Center of Shahid Mahallati Hospital, Tabriz, Iran; Department of Legal Medicine, AJA University of Medical Sciences, Tehran, Iran; Baqiyatallah University of Medical Sciences, Tehran, Iran; Department of Infectious Diseases, AJA University of Medical Sciences, Tehran, Iran

**Keywords:** Garlic, Low density lipoprotein cholesterol, High density lipoprotein cholesterol, Rat, Pharmacology

## Abstract

**Background:**

Hypercholesterolemia is associated with an increased risk of heart disease. In this study, we investigated the antihyperlipidemic effects of garlic (*Allium sativum* L.) in rat models of hypercholesterolemic.

**Methods:**

Wistar male rats were randomly divided into 4 diet groups with garlic supplementation. Male Wistar rats were fed by standard pellet diet (group I), standard diet supplemented with 4 % garlic (group II), lipogenic diet (containing sunflower oil, cholesterol and ethanol) equivalent to 200 mg raw garlic/kg body weight (raw) (group III) and lipogenic diet equivalent to 400 mg raw garlic/kg body weight (raw) (group IV).

**Results:**

Rats fed 400 g/kg garlic extract(GE), had a significantly lower concentration of serum low-density lipoprotein cholesterol (LDL-C) cholesterol and elevated HDL –C cholesterol at day 28 (*P* < 0.05).In addition,serum levels of LDL-C was lower in the III and IV group than those in the IV group (*P* < 0.001 for each). However, cholesterol efflux capacity was positively correlated with HDL cholesterol concentration (*P* < 0 · 0001). It was also directly correlated with garlic supplementation (*P* < 0 · 0001).

**Conclusion:**

Together Taken, the results are clearly indicative of the beneficial effects of garlic in reducing lateral side effects of hyperlipidemia. Our data demonstrate that GE has protective effects on HDL in rats with high LDL intake. Therefore, it could be used to remedy hypercholesterolemia with help reduce risk of coronary heart disease

**Virtual slides:**

The virtual slide(s) for this article can be found here: http://www.diagnosticpathology.diagnomx.eu/vs/1834155749171141

The article "High doses of garlic extract significantly attenuated the ratio of serum LDL to HDL level in rat-fed with hypercholesterolemia diet" was retracted in 2016. Reasons: plagiarism; compromised peer review; false authorship; unreliable data.

## Background

Hyperlipidemia is a major risk factor involved in ischemic heart disease. The prevalence of hyperlipidemia as well as its complications is increasing in the world. Moreover, alterations in serum lipid and lipoprotein levels result in a variety of chronic diseases such as coronary heart diseases (CHD) and atherosclerosis [1]. CHD is a major health problem in developed countries, and atherosclerosis is the principal contributor to the pathogenesis of myocardial and cerebral infarction [2], which in this case, there is convincing evidence that relaxation mediated by endothelium-derived nitric oxide (NO) is impaired in arteries from hypercholesterolemic and atherosclerotic animals [3, 4]. Many studies have now shown that elevated concentrations of total or LDL cholesterol in the blood are powerful risk factors for CHD [5], whereas high concentrations of HDL cholesterol or a low LDL (or total) to HDL cholesterol ratio may protect against CHD [2, 6].

Recent studies have directed their efforts toward the protective effects of plants such as garlic on hyperlipidemia [7, 8]. During the last few decades, the hypolipidemic effect of garlic and onion has been confirmed by many investigators, and many medications in the market that control hypercholesterolemia and hypertriglyceridemia. There have also been reports on the beneficial effects of garlic extract and oil in controlling hyperlipidemia in animals [7–13].

Garlic (*Allium sativum* L.) has long been used widely not only as a flavoring agent but also as a folk medication and is one of the most well-known herbal medicines worldwide and there has been increasing interest in using garlic as a cholesterol-lowering agent. Its reported beneficial actions and its compounds have been reported to have diverse biological activities such as cholesterol and triglyceride-lowering effects [14, 15],antimicrobial [16], antithrombotic [17], antihypertensive [18, 19] and anti-hyperlipidemic effects [20, 21],regulating plasma lipid levels, anti-carcinogenic, lead and mercury detoxification, antioxidant,, anti-diabetic, and various other biological actions [22–25]. Also, garlic has cardio-protective effects as it may help decrease TC, LDL- C and blood pressure while raising high HDL [26, 27]. The aim of this study was to evaluate of the anti-hyperlipidemic, and anti-hypercholesterolemic activities of garlic extract (GE) at doses of 200 and 400 mg/kg body weight for 2 and 4weeks, intraperitoneal (i.p.) prior to the induction of HDL/LDL, was investigated against hyperlipidemic/hypercholesterolemic in male rats

The article "High doses of garlic extract significantly attenuated the ratio of serum LDL to HDL level in rat-fed with hypercholesterolemia diet" was retracted in 2016. Reasons: plagiarism; compromised peer review; false authorship; unreliable data.

## Methods

### Animals and animal ethics/and or welfare

Forty healthy male Wistar albino rats weighing 200–250 grams were obtained from the Animal Care Center at College of Medicine, Shiraz University. Animals were housed in wire cages(four per cage,and rats were kept in individual propylene cages under standard laboratory conditions by the dimensions of 30 × 50 × 25 cm3 two by two,1 month before the start of the experiments, and maintained under a daily controlled lighting cycle(12 h-light and 12 h-dark) at 22 + 2 °C and 60 % humidity with free access to rat diet and tap water for one week to adapt to the laboratory environment prior to the experiments. Animals were kept for 4 weeks to allow acclimatization to the animal facility before starting the experiments.

All animals received human care according to the criteria outlined in the “Guide for the Care and Use of Laboratory Animals” prepared by the National Academy of Sciences and published by the National Institutes of Health

### Preparation of garlic extracts

Garlic bulbs utilized in these studies was purchased from a local grocery herb store in Shiraz, Iran. The garlic powder was prepared from fresh garlic bulb, which was heat-dried at 60–70 °C, and then ground by a mill. Volatile compounds in the garlic powder were analyzed by gas chromatography using daily disulfide as a standard [28, 29]. All garlic derivatives were stored at 4 °C and stocks of the water-soluble compounds were made fresh every time before use. Briefly, garlic cloves were peeled and homogenized with a small amount of quartz sand in 20 mmol/L Tris–HCl buffer (pH 7.4), and the debris was removed by centrifugation at 21,000 × g for 20 min at 25 °C. Subsequently, 30 g and 60 g of the powdered seeds were added to 400 ml and 800 ml of distilled water, and the extraction was obtained by steam distillation. The distillation process was continued until 200 mg/kg and 400 mg/kg of distillate were collected. The distillate was extracted three times with hydro-alcoholic liquid

### Experimental protocol/or procedure and treatments

The rats were divided into four groups and randomly allotted into one of four experimental groups each group contained ten animals. The control group was fed a standard diet (normal control)(for first stage 15 days and second stage 30 days) (n = 10), and test animals in group II was fed a standard diet plus 10 % cholesterol-enriched high-fat (U.A.R., Paris, France; hypercholesterolemic controls) (for 2 weeks and 4 weeks) (n = 10);

Groups III and IV, the rats were fed with a lipogenic diet containing standard pellet diet supplemented with 0.5 % (w/w) cholic acid, 20 % (w/w) sunflower oil and 2 % (w/w) cholesterol for at least two weeks to produce hyperlipidemia. Additionally, groups III and IV drank water containing 3 % (v/v) ethanol). Groups III and IV received garlic extract as an intraperitoneal (IP) dose of 200 and 400 mg/kg/bw (for 2 and 4 weeks) (garlic diet, n = 10), respectively. In addition, the garlic extract in experimental group was injected intraperitoneally. Blood samples were collected into test tubes containing EDTA through cardiac puncture. The plasma samples were separated by low speed centrifugation (2000 g) for 10 min and were stored at _80 _C until they were analyzed. All animal procedures were performed with regard to Iranian animal ethics society and local university rules.

The article "High doses of garlic extract significantly attenuated the ratio of serum LDL to HDL level in rat-fed with hypercholesterolemia diet" was retracted in 2016. Reasons: plagiarism; compromised peer review; false authorship; unreliable data.

### Plasma biochemical measurements/and or biochemical assay of serum lipids

Blood samples were taken directly from the heart in a centrifuge tube and allowed to form serum and processed as previously described, however, in each rat was determined after the start the treatment and every 15 d in total 2 times, and or can be expressed that after the 4-weeks treatment, the rats were killed using urethane anesthesia. The blood was collected by cardiac puncture and allowed to clot, and the clotted blood was then centrifuged at 4500 × g for 10 min. The serum was separated and stored at −80 °C for HDL and LDL analysis, and these serum concentrations were determined with commercially available enzyme kits (BioMerieux, Marcy, France).

### Statistical analysis

All data are presented as means ± SEM. Statistical analyses were analyzed using one-way ANOVA and two-way ANOVA, and significant differences between means were evaluated by the Tukey’s range post-hoc test compare between experimental groups. Differences with *P* < 0.05 were considered significant.

## Results

The effect of processed garlic on density lipoprotein-cholesterol characteristics is shown in Tables 1, 2, 3, 4, 5 and 6. After 2 and 4 weeks of treatment, LDL-c and HDL-c,decreased and increased significantly in the different groups, compared with control(I) and rats fed a diet enriched with high cholesterol groups(II),respectively, (P < 0.05).

**Table 1:** Effects of daily administration of garlic extract on plasma LDL profile for 2 and 4 weeks in male albino Wistar rats. The 95 % confidence interval of recalculated

Time	Groups	Mean ± SEM	Lower bound	Upper bound
2wk	Control	18.4000 ± 2.07364	15.8252	20.9748
2wk	hypercholesterolemic controls	25.8000 ± 1.48324	23.9583	27.6417
2wk	dose of 200 mg/kg/bw of garlic extract	21.8000 ± 8.22800	11.5836	32.0164
2wk	dose of 400 mg/kg/bw of garlic extract	19.2000 ± 3.49285	14.8631	23.5369
2wk	Total	85.2000 ± 2.87364	18.5075	22.3591
4wk	Control	11.4000 ± 4.33590	6.0163	16.7837
4wk	hypercholesterolemic controls	24.2000 ± 8.28855	13.9084	34.4916
4wk	dose of 200 mg/kg/bw of garlic extract	22.8000 ± 2.86356	19.2444	26.3556
4wk	dose of 400 mg/kg/bw of garlic extract	16.2000 ± 3.83406	11.4394	20.9606
4wk	Total	41.1000 ± 9.92418	15.3125	20.0342

The article "High doses of garlic extract significantly attenuated the ratio of serum LDL to HDL level in rat-fed with hypercholesterolemia diet" was retracted in 2016. Reasons: plagiarism; compromised peer review; false authorship; unreliable data.

**Table 2:** Effects of daily administration of garlic extract on plasma LDL profile for 2 weeks in male albino Wistar rats

Groups	Compared with groups	Mean difference (I-J)	Std. Error	Sig.	Lower bound	Upper bound
1	2	-.80000	2.49933	.999	−8.5278	6.9278
	3	4.00000	2.49933	.606	−3.7278	11.7278
	4	−7.40000	2.49933	.066	−15.1278	.3278
2	1	6.60000	2.49933	.126	−1.1278	14.3278
	3	11.40000	2.49933	.002	3.6722	19.1278
	4	7.40000	2.49933	.066	-.3278	15.1278
3	1	2.60000	2.49933	.899	−5.1278	10.3278
	2	3.40000	2.49933	.749	−4.3278	11.1278
	4	−4.00000	2.49933	.606	−11.7278	3.7278
4	1	−6.60000	2.49933	.126	−14.3278	1.1278
	2	.80000	2.49933	.999	−6.9278	8.5278
	3	4.80000^a^	2.49933	.415	−2.9278	12.5278

^a^Significant as compared to another groups

**Table 3:** Effects of daily administration of garlic extract on plasma LDL profile for 4 weeks in male albino Wistar rats

Groups	Compared with groups	Mean difference (I-J)	Std. Error	Sig.	Lower bound	Upper bound
1	2	4.8000	3.05666	.625	−14.2510	4.6510
	3	−5.24000*	3.05666	.526	−14.6910	4.2110
	4	−12.80000*	3.05666	.004	−22.2510	−3.3490
2	1	12.80000	3.05666	.004	3.3490	22.2510
	3	1.40000	3.05666	.997	−8.0510	10.8510
	4	8.00000	3.05666	.132	−1.4510	17.4510
3	1	11.40000*	3.05666	.012	1.9490	20.8510
	2	6.60000	3.05666	.293	−2.8510	16.0510
	4	−1.40000	3.05666	.997	−10.8510	8.0510
4	1	12.80000*	3.05666	.004	3.3490	22.2510
	2	8.00000	3.05666	.132	−1.4510	17.4510
	3	1.40000	3.05666	.997	−8.0510	10.8510

**Table 4:** Effects of daily administration of garlic extract on plasma HDL profile for 2 and 4 weeks in male albino Wistar rats. The 95 % confidence interval of recalculated

Time	Groups	Mean ± SEM	Lower bound	Upper bound
2wk	Control	41.4000 ± 3.64692	36.8718	45.9282
2wk	hypercholesterolemic controls	28.0000 ± 4.35890	22.5877	33.4123
2wk	dose of 200 mg/kg/bw of garlic extract	36.6000 ± .89443	35.4894	37.7106
2wk	dose of 400 mg/kg/bw of garlic extract	37.4000 ± 3.64692	32.8718	41.9282
2wk	Total	41.4000 ± 2.96463	34.7494	40.0506
4wk	Control	52.8000 ± 7.19027	43.8721	61.7279
4wk	hypercholesterolemic controls	29.6000 ± 9.39681	17.9323	41.2677
4wk	dose of 200 mg/kg/bw of garlic extract	31.4000 ± 4.33590	26.0163	36.7837
4wk	dose of 400 mg/kg/bw of garlic extract	33.2000 ± 3.27109	29.1384	37.2616
4wk	Total	82.5000 ± 7.20917	34.6368	42.9632

**Table 5:** Effects of daily administration of garlic extract on plasma HDL profile for 2 weeks in male albino Wistar rats

Groups	Compared with groups	Mean difference (I-J)	Std. Error	Sig.	Lower bound	Upper bound
1	2	13.40000	2.99333	.002	4.1448	22.6552
	3	4.80000	2.99333	.604	−4.4552	14.0552
	4	4.00000^a^	2.99333	.763	−5.2552	13.2552
2	1	−13.40000	2.99333	.002	−22.6552	−4.1448
	3	−8.60000	2.99333	.079	−17.8552	.6552
	4	−9.40000^a^	2.99333	.045	−18.6552	-.1448
3	1	−4.80000	2.99333	.604	−14.0552	4.4552
	2	8.60000	2.99333	.079	-.6552	17.8552
	4	-.80000	2.99333	1.000	−10.0552	8.4552
4	1	−4.00000^a^	2.99333	.763	−13.2552	5.2552
	2	9.40000**	2.99333	.045	.1448	18.6552
	3	8.0000	2.99333	1.000	−8.4552	10.0552

^a^Significant as compared to another groups

The article "High doses of garlic extract significantly attenuated the ratio of serum LDL to HDL level in rat-fed with hypercholesterolemia diet" was retracted in 2016. Reasons: plagiarism; compromised peer review; false authorship; unreliable data.

**Table 6:** Effects of daily administration of garlic extract on plasma HDL profile for 4 weeks in male albino Wistar rats

Groups	Compared with groups	Mean difference (I-J)	Std. Error	Sig.	Lower bound	Upper bound
1	2	23.20000	3.97240	.000	10.9176	35.4824
	3	21.40000*	3.97240	.000	9.1176	33.6824
	4	19.60000*	3.97240	.001	7.3176	31.8824
2	1	−23.20000	3.97240	.000	−35.4824	−10.9176
	3	−1.80000*	3.97240	.997	−14.0824	10.4824
	4	−3.60000*	3.97240	.941	−15.8824	8.6824
3	1	−21.40000*	3.97240	.000	−33.6824	−9.1176
	2	−19.60000*	3.97240	.001	−31.8824	−7.3176
	4	1.80000	3.97240	.997	−10.4824	14.0824
4	1	−19.60000*	3.97240	.001	−31.8824	−7.3176
	2	−17.80000*	3.97240	.002	−30.0824	−5.5176
	3	1.80000	3.97240	.997	−10.4824	14.0824

### Plasma lipid profiles of LDL-c level

First stage; between 1–15 days (2 weeks): Tables 1 and 2 shows that between groups 2 and 4 induced a significant increase in serum LDL-C (*P* <0/05) and a significant decrease in the serum LDL-C level in comparison with the control. Also, between 3 and 4, there is a significant difference (*P* <0/05) and showed a significant decrease in serum LDL-C level, when compared to that of groups I and II (Fig. 1)(Tables 1 and 2).

**Fig. 1:** Effect of garlic extracts (200 and 400 mg/kg) on serum LDL levels in comparison with the control and hypercholesterolemic groups for 2 weeks on the activity of LDL. Note that statistically significant difference from the control group with other groups. *Significant as compared to 200 mg/kg group. Bars are expressed as mean ± SEM (n = 10). *P* < 0.05

Second stage; between 1–30 days (4 weeks): Tables 1 and 3 reveals a significant decrease of serum LDL-C level between groups 1 and 4 (*P* <0/05). Furthermore, this significant decrease in between groups 1 and 2, 1 and 3, 1 and 4 were observed in groups fed the processed garlic-supplemented diet (*P* <0.05), so the plasma LDL in treated groups decreased significantly, compared with those of I and II groups. Finally, LDL-cholesterol did show significant change and, demonstrating that dietary supplementation with processed garlic improved lipid profiles (Fig. 2)(Tables 1 and 3).

The article "High doses of garlic extract significantly attenuated the ratio of serum LDL to HDL level in rat-fed with hypercholesterolemia diet" was retracted in 2016. Reasons: plagiarism; compromised peer review; false authorship; unreliable data.

**Fig. 2:** Effect of garlic extracts (200 and 400 mg/kg) on serum LDL levels in comparison with the control and hypercholesterolemic groups for 4 weeks on the activity of LDL. Note that statistically significant difference from the control group with other groups . Bars are expressed as mean ± SEM (n = 10). *P* < 0.05

### Plasma lipid profiles of HDL-c level

First stage; between 1–15 days (2 weeks): Table 4 and 5 indicates that between groups 1 and 2, 2 and 4, 5 and 6 created a significant increase in serum HDL-C (*P* <0/05) and a significant increase in the serum HDL-C level in comparison with I and II groups,the other expression, serum levels of HDL-cholesterol were also increased in the garlic supplemented group compared to those in the control group, there was statistically significant difference in lipid profile among various groups at the beginning of the study. A significant (*p* <0.05) increase in the level of HDL was observed on IP administration of HDL-c. By comparing the different animal groups, it was observed that rats which received garlic extracts showed the utmost reduction in serum HDL-C levels compared to those which received garlic alone (Fig. 3) (Tables 4 and 5).

**Fig. 3:** Effect of garlic extracts (200 and 400 mg/kg) on serum HDL levels in comparison with the control and hypercholesterolemic groups for 2 weeks on the activity of HDL. Note that statistically significant difference from the control group with other groups . Bars are expressed as mean ± SEM (n = 10). *P* < 0.05

Second stage; between 1–30 days (4 weeks): Table 4 and 6 demonstrates that between groups 2 and 3, 2 and 4, as well as groups 1 and 3, 2 and 3 a significant increase in serum HDL-C in comparison with I and II groups (*P* <0/05). In total, in treated group, a significant increase (*p* < 0.05) in serum HDL levels was detected compared to I and II groups. To warp up, the test group had significantly lower plasma concentrations of LDL-C, in comparison with I and II group. While the HDL-C level was significantly increased in the treated group with garlic in comparison with rats fed a high-fat diet. Our results suggest that administration of high doses of garlic extracts shows protective effects on HDL in rats with high LDL intake (Fig. 4)(Tables 4 and 6).

**Fig. 4:** Effect of garlic extracts (200 and 400 mg/kg) on serum HDL levels in comparison with the control and hypercholesterolemic groups for 2 weeks on the activity of HDL. Note that statistically significant difference from the control group with other groups.* Significant as compared to control group with treatment groups. Bars are expressed as mean ± SEM (n = 10). *P* < 0.05

The article "High doses of garlic extract significantly attenuated the ratio of serum LDL to HDL level in rat-fed with hypercholesterolemia diet" was retracted in 2016. Reasons: plagiarism; compromised peer review; false authorship; unreliable data.

## Discussion

Natural remedies have been investigated for centuries for a wide variety of ailments. Among them, garlic has received special attention for its beneficial effects [30–36]. Common available garlic preparations in the form of garlic oil, garlic powder and pills are widely used for certain therapeutic purposes, including lowering blood pressure and improving lipid profile [37–39]. Despite the impressive effects of garlic, most studies are limited by lack of controlled methods and by the use of reparations with unknown amounts and chemical identification of the active ingredient. Therefore this study was designed to examine the effects of raw and boiled garlic and their aqueous extracts on lipid, antioxidant and protein status in serum of rats. For this purpose, Wistar rats were fed diets with garlic and cholesterol supplements.

This study has shown that administration of 200 mg/kg/bw, especially 400 mg/kg/bw dietary garlic significantly attenuated serum LDL levels and increased HDL levels in when fed 1 % cholesterol in the fed rats. The significant reduction in the ratio of LDL to HDL/LDL with garlic suggests potential health benefits of garlic supplementation in reduction of coronary artery disease and/or atherosclerosis and/or similar to those described in the field malignant cholesterol diseases. Our findings were in agreement with other studies, which announced that garlic consumption increased HDL-C level in hyperlipidemic patients [7], animals [40], and patients with coronary artery disease [41]. When garlic supplements was added into the diet at a concentration of 1 %, LDL-C level was decreased and HDL-C level were increased in rabbits [42], resulting in a decrease in the LDL-C/HDL-C ratio. Moreover, our observations reveal that the dietary garlic extracts may have cardiovascular diseases protection effects by regulating the LDL-C/HDL-C ratio.

Furthermore, *in vivo and in vitro* studies in recent years have demonstrated that garlic has cholesterol and triglyceride-lowering, antibacterial, hypoglycemic, hypotensive potential and anti-aggregatory properties [24, 43–45]. The effects of garlic on serum lipid levels have been investigated in human and animal models and indicate inconsistency in the reported results [46],which according to these findings can be expressed that our results is exactly in agreement with those mentioned. and, when compared to groups I and II, the significant improvement of lipid profiles in group III and IV rats treated simultaneously with garlic extracts agrees with the previous studies that garlic is a hypolipidemic agent [47] that can help in decreasing the level of LDL-C and in increasing the level of HDL-C. In parallel to, in hypertensive patients, Durak *et al.* reported that garlic extract supplementation improves blood lipid profile, strengthens blood antioxidant potential and decreases the level of malondialdehyde in blood samples [48], and also, another study by Bordia *et al.*, showed that in patients suffering from coronary artery disease, administration of garlic significantly decreased serum LDL and increased HDL[41]. In a human study, supplementation with raw garlic, powdered garlic, or aged garlic extract (4 g/day) for 6 months significantly lowered LDL-C and other plasma lipid levels in adults with moderate hypercholesterolemia [49]. Our findings in rats provide further support for the anti-hyperlipidemic, and anti-hypercholesterolemic of processed garlic products and garlic exhibited remarkable anti-hyperlipidemic action by decreasing the levels of LDL-C in plasma for groups control and % 1 fed with cholesterol diet and increasing the level of HDL for groups with doses 200 mg/kg and 400 mg/kg, respectively. Although significant reductions in blood cholesterol and triglyceride levels were found in some studies when garlic extract or powder were utilized, no satisfactory agreement has been reached on this kind of clinical and experimental data[49].

The article "High doses of garlic extract significantly attenuated the ratio of serum LDL to HDL level in rat-fed with hypercholesterolemia diet" was retracted in 2016. Reasons: plagiarism; compromised peer review; false authorship; unreliable data.

## Conclusions

In conclusion, the high doses of garlic extracts ameliorated plasma lipid profiles by decreasing the LDL-C level and increasing the HDL-C level in high-fat fed rats. Therefore, our findings revealed that the garlic extract treatment can lower blood cholesterol level, such as LDL and can improve blood lipid profile to a significant extent, such as HDL. Finally, it has been recommended that extracts such as garlic that are rich in anti-hyperlipidemic, and anti-hypercholesterolemic contents may confer beneficial effects in this regard to atherosclerotic processes.
